RETRACTED

# CT Image Features of the FBP Reconstruction Algorithm in the Evaluation of Fasting Blood Sugar Level of Diabetic Pulmonary Tuberculosis Patients and Early Diet Nursing

**DOI:** 10.1155/2021/1101930

**Published:** 2021-11-18

**Authors:** Lili Hong, Liling Lin, Jingping Chen, Biyu Wu

**Affiliations:** ^1^Pulmonary and Critical Care Medicine (PCCM), Quanzhou First Hospital, Quanzhou, 362000 Fujian, China; ^2^Hospital Infection-Control Office, The Second Affiliated Hospital of Fujian Medical University, Quanzhou, 362000 Fujian, China; ^3^Department of Nursing, Quanzhou First Hospital, Quanzhou, 362000 Fujian, China

## Abstract

The study was aimed at exploring the application value of the CT image based on a filtered back projection (FBP) algorithm in the diagnosis of patients with diabetes complicated with tuberculosis and at analyzing the influence of dietary nursing on patients with diabetes complicated with tuberculosis. In this study, the FBP algorithm was used to optimize CT images to effectively obtain reconstructed ROI images. Then, the deviation from measurement values of reconstructed images at different pixel levels was analyzed. 138 patients with diabetes complicated with tuberculosis were selected as research subjects to compare the number of lung segments involved and the CT imaging manifestations at different fasting glucose levels. All patients were divided into the control group (routine drug treatment) and observation group (diet intervention on the basis of drug treatment) by random number table method, and the effect of different nursing methods on the improvement of patients' clinical symptoms was discussed. The results showed that the distance measurement value decreased with the increase in pixel level, there was no significant difference in the number of lung segments involved in patients with different fasting glucose levels (*P* > 0.05), and there were statistically significant differences in the incidence of segmental lobar shadow, bronchial air sign, wall-less cavity, thick-walled cavity, pulmonary multiple cavity, and bronchial tuberculosis in patients with different fasting glucose levels (*P* < 0.05). Compared with the control group, 2 h postprandial blood glucose level in the observation group was significantly improved (*P* < 0.05), there was a statistical significance in the number with reduced pleural effusion and the number with reduced tuberculosis foci in the two groups (*P* < 0.05), and the level of hemoglobin in the observation group was 7.1 ± 1.26, significantly lower than that in the control group (8.91 ± 2.03, *P* < 0.05). It suggested that the changes of CT images based on the FBP reconstruction algorithm were correlated with fasting blood glucose level. Personalized diet nursing intervention can improve the clinical symptoms of patients, which provides a reference for the clinical diagnosis and treatment of patients with diabetes complicated with tuberculosis.

RETRACTED

## 1. Introduction

Diabetes and tuberculosis are common diseases, and their long-term existence will cause chronic damage or failure of multiple organs [1, 2]. According to statistics, the prevalence of tuberculosis in diabetic patients is 4 to 8 times higher than that in the general population. The metabolism disorder of sugar, fat, and protein in diabetic patients leads to a decline in immunity, and the increased blood sugar provides nutrition for the growth and reproduction of mycobacterium. As a result, the diabetic patients are easy to develop tuberculosis [3–5]. Of diabetic patients suffering from tuberculosis, approximately 10%-20% of patients have no respiratory symptoms, and about 80% of patients have rapid onset and disease progress, poor curative effects, and a high drug resistance rate [6]. Compared with simple pulmonary tuberculosis, the scope of lung lesions is wide and there are many caseous lesions, and thus, the treatment is difficult and the prognosis is poor [7, 8]. At present, the clinical treatment of diabetes patients with tuberculosis is mainly the drug treatment and diet intervention to control the patient's blood glucose level [9, 10].

The examination methods of diabetes complicated with tuberculosis mainly include X-ray and CT, but the X-ray is inferior to CT in determining the activity of tuberculosis [11]. Multislice spiral CT overcomes the image overlap problem in traditional X-ray examinations thanks to its high density and spatial resolution and significantly increases the detection rate of lesions. However, its images show variability and complexity when diagnosing atypical diseases such as diabetes and tuberculosis [12, 13]. CT images of patients with diabetes and tuberculosis mostly show segmental and leaf-shaped lesions, consolidation, and cavities formed by the dissolution and necrosis of caseous material, and the cavity is connected to the surrounding bronchus [14, 15]. After effective treatment, the CT image shows that the scope of the lesion is reduced and the exudative boundary becomes clear, but there exist a few cord-like and irregular thin-line shadows [16, 17].

The data obtained by the CT system in the two-dimensional plane is processed, there will inevitably be errors in the installation process, and it needs to be calibrated through the template. Some scholars have proposed CT image iterative reconstruction algorithms, FBP algorithms, and quantitative analysis of optical tomography molecular imaging to analyze the quality of image reconstruction under different filters and sparseness. The FBP algorithm has the characteristics of simple operation and short running time when processing CT images, but it has the problem of high radiation dose and needs to be further optimized [19]. In order to reduce the harm of X-rays to the human body, the CT image is reconstructed, the ROI projection data is used to increase or decrease the projection data of the region of interest (ROI), and the constructor is used to reconstruct the overall or partial image [20]. For the convolutional backprojection calculation of image reconstruction, the ROI area can be selected, and it is not necessary to scan the whole to obtain all the projection data [21, 22]. Based on the above research, in this study, the FBP algorithm was used to reconstruct CT images, and different ways of nursing were adopted in the two groups, to discuss the influence of different nursing methods on the patient condition, expected to provide a basis for the diagnosis and treatment of diabetes complicated with tuberculosis.

RETRACTED

## 2. Materials and Methods

### 2.1. Research Subjects

In this study, 138 patients with diabetes and tuberculosis admitted to hospital from June 2017 to January 2021 were selected as research subjects, including 71 males with an average age of 45.6 ± 7.1 years and 67 females with an average age of 46.4 ± 8.5 years. A random number table method divided them into the observation group and control group, with 69 cases in each group. The control group was given conventional treatment, and the observation group was given dietary intervention on the basis of drug treatment. There were 35 males and 34 females in the control group, with an average age of 45.47 ± 5.18 years; there were 36 males and 33 females in the observation group, with an average age of 46.02 ± 6.23 years. The study has been approved by the ethics committee of the hospital. All patients and their families were aware of the study and had signed an informed consent form.

Inclusion criteria were as follows: (1) patients aged ≥18 years old and no limitation to the gender and (2) patients diagnosed with diabetes and tuberculosis.

Exclusion criteria were as follows: (1) patients with AIDS and other diseases that affect the immune system, (2) patients with a history of insulin treatment, (3) patients with vital organ dysfunction, and (4) patients with endocrine diseases and severe gastrointestinal dysfunction.

### 2.2. CT Imaging

X-ray is a way for CT to obtain information on the internal structure of the human body. The most important way is to use a detector to capture the attenuated X-rays passing through the human body. The acquisition of CT images is mainly to use algorithm reconstruction to reconstruct the projection data acquired by the detector at different angles. In the medical field, the basic unit of CT reconstruction is generally voxels. Voxels divide the tissue into small blocks with uniform density, and the resulting uniform blocks are called voxels. The finer the division of the tissue, the smaller the voxel, which means that the interval between the receivers on the detector is also smaller. For the same object, the detector can obtain more projection data, and the quality of the reconstructed image becomes better. The data flow chart of CT system imaging is shown in Figure 1. First, the X-ray tomographic plane is concealed. The X-ray on the X-ray receiver is the projection data to collect, and the collected information reconstructs the image information (Figure 1).

RETRACTED

### 2.3. Optimization of the FBP Algorithm

The projection process equation of the *A* × *A* size two-dimensional image is as follows: *D* = *QH* (1), where *H* represents the image vector of size *AA* × 1, *Q* represents the projection coefficient matrix of *YW* × *AA* (*W* represents the projection angle and *Y* represents the maximum number of projections at each projection angle), and *D* represents the projection vector of size *YW* × 1. The reconstructed image is shown in

(1) $$\begin{array}{c} B*=Q*D. \end{array}$$

In the equation, *B*∗ is the reconstructed image with a size of *AA* × 1 and *Q*∗ represents the generalized inverse of the projection coefficient matrix *Q*. The calculation of *Q*∗ directly will be slightly complicated and consume reconstruction time. It can be replaced by other calculations, which can save computing time. According to the following principles, the first-order iterative method is used to obtain *Q*∗.

If the initial estimate of the generalized inverse *Q*∗ of the projection coefficient matrix *Q* of *YW* × *AA* is set to *N*_0_, set the residual *S*_0_ = *D*_R(*T*)_ − *QN*_0_ to meet *γS*_0_ < 1, where *γS*_0_ represents the spectral radius of *S*_0_ and *D*_R_(*Q*) is the orthogonal matrix of *Q*; then, the sequence [*N*_0_, *N*_1_ ⋯ ⋯*N*_*K*_, *N*_*K*+1_, ⋯⋯] can be expressed by

(2) $$\begin{array}{c} NK+1=Nk+N0-N0QNK,\;K=0,1\cdots \cdots . \end{array}$$

When *K*⟶∞, the equation converges to *Q*∗; then, the corresponding sequence of the residual value meets the requirements of the following equation.

(3) $$\begin{array}{c} ║S_{K+1}║\leq ║S_{0}║S_{K}║,\;\;K=0,1,\cdots \cdots . \end{array}$$

The norm of any multiplication matrix conforms to *S*_*K*_ = *D*_R(*T*)_ − *QN*_*K*_.

In order to facilitate the approximate value *N*_0_ of the initial value of *Q*∗, simply consider it equal to

(4) $$\begin{array}{c} N_{0}=\theta Q^{t}. \end{array}$$

In the equation, *Q*^*t*^ is the transposition of *Q* and *θ* is an actual value and conforms to the following equation:

(5) $$\begin{array}{c} 0<\theta <\frac{2}{\lambda 1\;\left({QQ}^{t}\right)}. \end{array}$$

In the equation, *λ*1 (*QQ*^*t*^) is the largest nonzero eigenvalue of *QQ*^*t*^.

RETRACTED

In order to avoid the difficulty of calculating the relatively large values of *Q* and *Qq*, both sides of the equation in equation (3) are multiplied by the projection value *D* at the same time, and we get

(6) $$\begin{array}{c} N_{K+1}D=N_{K}D+N_{0}D-N_{0}{QN}_{K}D,\;K=0,1\cdots \cdots . \end{array}$$

*N*_*K*+1_ *D* and *N*_*K*_*D* represent the *K* + 1 and *K*th reconstructed images *H*^*i*^_*K*+1_ and *H*^*i*^_*K*_, *N*_0_*D* is the initial image *H*^*i*^_0_, and *N*_0_*QN*_*K*_*D* represents the projection of *H*^*i*^, and finally, the reconstruction is performed. The FBP algorithm is used to reconstruct the image. *θ* times to replace *N*_0_*QN*_*K*_*D*. When *AA* < *YW*, *θ* = 1; when *NN* > *YW*, *θ* < 2^−*AA*/*YW*^. Equation (6) can be simplified as follows.

(7) $$\begin{array}{c} H_{K+1}^{i}=H_{K}^{i}+H_{0}^{i}-N_{0}QH_{K}^{i}. \end{array}$$

In order to verify the performance of the algorithm, the following experiments are carried out (Figure 2). In the experiments, the value of *θ* is all 1.

### 2.4. Algorithm Steps

According to the principle of the algorithm, the steps of the algorithm as shown in Figure 3 are as follows: first, the first step is to initialize *θ* and the termination condition *φ*.

In the second step, when *K* = 0, the FBP algorithm reconstructs the image Hifbp to obtain the preprocessed image *H*^*i*^_0_ = *θH*^*i*^_flp_.

The third step is to project *H*^*i*^_*K*_ to obtain the projection value *D*_*k*_.

The fourth step is to reconstruct the image according to *D*_*k*_ according to FBP and multiply the result obtained by *θ* to obtain *H*_*r*_.

The fifth step is to correct the image, and the equation is *H*^*i*^_*K*+1_ = *H*^*i*^_*K*_ + *H*^*i*^_0_ − *H*^*i*^_*r*_.

In the sixth step, make Δ = ║*H*^*i*^_*K*+1_ − *H*^*i*^_*K*_║≤*K* = *k* + 1; in the last step, if Δ > *φ*, it will return to step three; otherwise, the loop will end.

### 2.5. Test Inspection Method

1. CT scanning method: the patients participating in the study were all in an empty stomach state before the examination, and they were allowed to drink moderately before the examination. Using the Philips 16-slice spiral CT scanner, the patient was placed in a supine position and the chest was scanned axially from the lung tip to the top of the diaphragm. The scanning parameters are as follows: select reconstruction layer thickness 8 mm, reconstruction layer distance 8 mm, tube voltage 100~150 kV, and tube current 30~45 mA, combined with the scanned image results, select a multiangle, and carefully observe in a multidirectional manner and reconstruct the present image. All patients received the first multislice spiral CT scan within 5 days, the data that appeared for the first time were reconstructed by an iterative algorithm, and the sensitive parts of the patient were protected during each scan. After the scan, the two attending radiologists will read and analyze the pictures
2. Then, 0.5 mL of median cubital venous blood was collected from each patient under fasting and transferred to a sterile blood collection tube with 50 *μ*L of heparin. After centrifugation, the upper plasma was collected and tested with an automatic biochemical analyzer

RETRACTED

### 2.6. Statistical Methods

The data in this study were sorted out using Excel 2019 and processed by SPSS 22.0. The measurement data were expressed as $\bar{x}\pm s$, and the count data was expressed as a percentage (%). If the data between groups obeyed the normal distribution, the *t*-test was used; if not, the rank sum test was used, and *α* = 0.05 was used as the test standard. *P* < 0.05 indicated that the difference was statistically significant.

## 3. Results

### 3.1. The Image of the Algorithm

In the case of using the same dose in Figure 4, it can be seen that the noise of the Figure 4(b) image is relatively large and the graininess is strong. After the Figure 4(a) image uses the FBP reconstruction algorithm for noise processing, the image definition is higher, the image noise level is greatly improved, and the smoothness of the image is improved.

### 3.2. Video Image

The iterative reconstruction algorithm reconstructs the image based on the estimation of the statistical model of the observation data.  Figure 5(a) is the imaging result of the FBP reconstruction algorithm.  Figure 5(b) shows the marked part in Figure 5(a). The FBP reconstruction algorithm can extract image features well (Figure 5).

### 3.3. Error Comparison of Different Boundary Pixels

For the same local area, 4, 6, and 8 pixels were selected to compare the measured values of FBP reconstruction in the ROI. At different pixel numbers, different distance measurement values will be obtained. As the number of local data increases, the smaller the distance measurement value, the smaller the error obtained, which means that the more local data are selected, the better the ROI reconstruction obtained and the better the image effect (Figure 6).

RETRACTED

### 3.4. CT Detection Results of Fasting Blood Glucose Levels in Patients

All patients accepted examinations for the fasting blood glucose level. As per the *Guidelines for Prevention and Treatment of Type 2 Diabetes in China*, the 138 patients were divided into the good blood glucose level group (<7 mmol/L), normal blood glucose level group (7-10 mmol/L), and poor blood glucose group (>10 mmol/L), as shown in Figure 7. There was no statistical difference in the age, the average duration of tuberculosis, and the average duration of diabetes (*P* > 0.05).

The results are shown in Figure 8. Patient 1 was a 62-year-old male. CT examination suggested multiple lung infections. The lesions concentrated on the left upper lobe and right lower lobe, accompanied by multiple cavities and a small amount of bilateral pleural effusion (Figures 8(a)–8(c)). Patient 2 was a 60-year-old male. CT examination showed exudative lesions in both lungs and multiple cavities in the upper right and lower left lungs, suggesting bilateral lung infection (Figures 8(d)–8(f)). Patient 3 was a 54-year-old female, and the CT examination showed pulmonary tuberculosis in the upper left lung, accompanied by cavitation and mediastinal lymph node calcification (Figures 8(g)–8(i)).

CT examination of the most frequent sites of lesions in patients with diabetes and tuberculosis showed that the average number of lung lesions involved in patients with good fasting blood glucose levels was 5.8 ± 3.9, that in patients with normal fasting blood glucose levels was 6.0 ± 4.1, and that in patients with poor fasting blood glucose levels was 6.1 ± 3.8. There was no significant difference in the number of lung lesions involved in patients with different fasting blood glucose levels (*P* > 0.05) (Figure 9).

CT images of patients with diabetes and pulmonary tuberculosis usually showed segmental, large lobular fusion lesions and consolidation, cavitation, pleural effusion, and lymph node enlargement. Then, the relationship between different fasting blood glucose levels and the imaging manifestations was analyzed. The results showed that of the 25 patients with good fasting blood glucose levels, 14 had three-segment large leaf-like shadows, 18 had proliferative nodular shadows, 11 had bronchial inflation signs, 7 had wall-less cavities, 7 had thick-walled cavities, 8 had multiple cavities in the lungs, 4 had thin-walled cavities, and 6 had bronchial tuberculosis. Of 41 patients with normal fasting blood glucose levels, 25 cases had three-segment leaf-like large shadows, 30 cases developed proliferative nodular shadows, 22 cases had bronchial inflation signs, 15 cases had wall-less cavities, 14 cases had thick-walled cavities, 17 cases had multiple cavities in the lungs, 7 cases had thin-walled cavities, and 14 cases had bronchial tuberculosis. Of 72 patients with poor fasting blood glucose levels, 57 cases had three-segment leaf-like large shadows, 53 cases had proliferative nodular shadows, 55 cases had bronchial inflation, 36 cases had wall-less cavities, 35 cases had thick-walled cavities, 40 cases had multiple cavities in the lungs, 12 cases had thin-walled cavities, and 35 cases had bronchial tuberculosis.  Figure 10 shows the incidence of eight types of imaging manifestations with different fasting blood glucose levels. The results showed that there was no significant difference in the incidence of proliferative nodules and thin-walled cavities in patients with different fasting blood glucose levels (*P* < 0.05), but segmental leaf-like large-scale shadows, bronchial inflation sign, wall-less cavities, thick-walled cavities, multiple cavities in lungs, and the incidence of bronchial tuberculosis showed statistically significant differences (*P* < 0.05).

RETRACTED

### 3.5. Comparison of the Effects of Dietary Intervention between the Two Groups of Patients

After 138 patients were randomly divided into groups, the effects of dietary intervention on the various indicators of the patients were analyzed. The results showed that in the observation group, the glucose level was 11.32 ± 1.48 mmol/L 2 h after meal and it was 14.55 ± 1.87 mmol/L in the control group. Compared with the control group, the observation group's blood glucose level 2 h after meal improved significantly, and the difference was statistically significant (*P* < 0.05). After diet intervention, it was found that in the observation group, the pleural effusion was significantly reduced in 61 patients and the tuberculosis lesions of 51 patients were significantly reduced; in the control group, the pleural effusion of 32 patients was significantly reduced and the tuberculosis lesions of 27 patients were significantly reduced. The difference was statistically significant in terms of the number of lesions reduced (*P* < 0.05). The hemoglobin level in the observation group after intervention was 7.1 ± 1.26, and that in the control group was 8.91 ± 2.03; the difference was statistically significant (*P* < 0.05) (Figure 11).

## 4. Discussion

Diabetes is a chronic metabolic disease. Due to metabolic disorder and low immunity, the patients are susceptible to tuberculosis. Diabetes complicated with tuberculosis develops rapidly, and the lesions are widely distributed and easy to form cavities, which makes it difficult to treat [23]. The treatment and prognosis of diabetes with pulmonary tuberculosis depend to a certain extent on the degree of blood glucose control. A reasonable diet can provide patients with sufficient nutrition and avoid hyperglycemia. Therefore, the patient's fasting blood glucose level can be used as a blood glucose detection indicator [24]. To prevent the drug and food intake from interacting with blood sugar levels which will affect the clinical treatment, it is a must that patients undergo regular chest examinations. Diabetes and tuberculosis lesions with different levels of fasting blood glucose may have different CT manifestations.

RETRACTED

The choice of a CT contrast agent is related to the detection ability of the lesion and the early clinical diagnosis rate of the disease. Compared with single-slice spiral CT, multislice spiral CT has multiple rows of detectors, which not only increases the scanning speed but also shortens the time of one revolution to 0.5 s. It can also obtain multilayer images during one revolution. Because it is a fast volume scan, it is possible to conduct uninterrupted data collection on a large area of the body in a short time, and the information obtained can also be increased. After computer processing, the imaging of multiple technologies is completed, and the image quality is higher. The virtual endoscopy not only is more real but also improves the detection rate of smaller lesions and mucosal lesions. On this basis, the image is reconstructed by the FBP algorithm, which can effectively improve the image quality. The reconstruction algorithm divides the entire image processing process into many times and gradually improves the image processing. In most low-dose scans, the scanned image processing parameters must be optimized to maximize the image quality. Algorithms and various noise reduction techniques can achieve the effect of smoothing the image [25]. The FBP algorithm is applied to low-dose CT images for denoising, iterative reconstruction, image postprocessing, and sinusoidal image preprocessing; the FBP algorithm can denoise low-dose CT images, which is consistent with the results of this study. This study also used low-dose scans, and the results showed that the FBP reconstruction algorithm showed good superiority in lung CT imaging scans. After the image is reconstructed by the iterative algorithm, the image quality and image information are significantly improved. For the same local area, compare the measured value of the FBP reconstruction in the ROI. The more the number of local data in the image, the smaller the distance measurement value and the smaller the error. That is to say, the more local data are selected, the better the effect of the ROI reconstruction image. In this study, the relationship between fasting blood glucose and CT findings in patients with diabetes and pulmonary tuberculosis was detected. The results showed that due to the existence of multiple pathological properties, the CT imaging of patients showed coexistence of multiple morphological and dense lesions. Because a large number of mycobacterium invaded the patient's lung tissue, it caused changes in the CT imaging of the patient's lung. The exit rate also increases, which is consistent with research results of Barreda et al. [26].

RETRACTED

The bronchial inflation symptom reflects the inflammatory lesions of patients. This study found that as the fasting blood sugar level of patients increased, the incidence of bronchial inflation syndrome also increased. Cavitation is an important pathological feature of active tuberculosis. The results of this study showed that the incidence of wall-less cavities, thick-walled cavities, and multiple pulmonary cavities increased with the increase in the patient's fasting blood glucose level. Additionally, the incidence of bronchial tuberculosis also increased. This was in line with the results of Xia et al. [27]. The main cause may be the necrosis and liquefaction of the caseous material in the small bronchus, and the drainage bronchus and substances containing tubercle bacilli adhere to the inner wall of the bronchus and cause local infection in the patient. After diet intervention, it was found that in the observation group, blood glucose levels, pleural effusion, tuberculosis lesions, and glycosylated hemoglobin levels improved significantly 2 h after meals, indicating that diet nursing intervention positively affected blood glucose control in patients with diabetes and tuberculosis.

## 5. Conclusion

In this study, the FBP reconstruction algorithm was applied to CT images of patients with diabetic tuberculosis, and the relationship between fasting blood glucose levels and CT imaging findings in patients with diabetes and tuberculosis was detected. Finally, the effect of diet intervention on the improvement of clinical symptoms of patients was analyzed. The results show that the CT image definition of the PDF reconstruction algorithm is relatively high, and the image has good classification characteristics. The more local data of the image are selected, the better the ROI reconstruction image obtained and the better the CT image effect. The fasting blood glucose level is closely related to the patient's CT manifestations. The change of fasting blood glucose level will cause changes in CT imaging. Through personalized diet nursing intervention, the patient's blood glucose can be controlled to a certain extent and clinical symptoms can be improved, which has a certain clinical promotion value.

RETRACTED

## Figures and Tables

**Figure 1:** Schematic diagram of the data flow of CT system imaging.

**Figure 2:** Flow chart of the reconstruction algorithm principle.

**Figure 3:** Flow chart of algorithm steps.

**Figure 4:** Comparison of low-dose lung original image and reconstruction algorithm: (a) CT image reconstructed by the FBP algorithm; (b) original CT image.

**Figure 5:** Image reconstruction algorithm feature label map of the lungs: (a) CT image reconstructed by the FBP algorithm; (b) the marked part in (a).

**Figure 6:** Distance measurement values of different pixel reconstruction results. ∗ represents a statistical difference compared with pixel 8 (*P* < 0.05).

**Figure 7:** Comparison of basic data of patients with different blood glucose levels: (a) gender; (b) average age; (c) average duration of tuberculosis; (d) average duration of diabetes.

**Figure 8:** CT examination results of patients with diabetes and pulmonary tuberculosis.

**Figure 9:** Comparison of the number of lung lesions involved in different fasting blood glucose levels.

**Figure 10:** The incidence of CT imaging manifestations in patients with different fasting blood glucose levels.

**Figure 11:** Comparison of various indicators between the two groups of patients after intervention.

## Data Availability

The data used to support the findings of this study are available from the corresponding author upon request.
